# MicroRNA-200c as a prognostic and sensitivity marker for platinum chemotherapy in advanced gastric cancer

**DOI:** 10.18632/oncotarget.17087

**Published:** 2017-04-13

**Authors:** Min Li, Kangsheng Gu, Wei Liu, Xiaoque Xie, Xiaolu Huang

**Affiliations:** ^1^ Department of Oncology, The First Affiliated Hospital of Anhui Medical University, Hefei, Anhui 230022, P.R. China; ^2^ Department of Oncology, Huaibei People's Hospital, Huaibei, Anhui 235000, P.R. China

**Keywords:** miR-200c, gastric cancer, chemotherapy

## Abstract

We examined microRNA-200c (miR-200c) expression in tumor tissues and plasma of patients with advanced gastric cancer and correlated miR-200c expression with treatment efficacy of platinum chemotherapy and patient prognosis. Tumor tissues were collected from 51 patients with advanced gastric cancer who received platinum-containing chemotherapies. The plasma was collected from the same group of patients and 51 subjects with chronic superficial gastritis. Quantitative RT-PCR was used to evaluate miR-200c expression, and its correlation with treatment efficacy and patient prognosis was analyzed.

The results showed that the miR-200c expression in gastric cancer tissues and in plasma were significantly lower than tumor-adjacent tissues and in patients with chronic superficial gastritis (both *p <*0.05). No significant correlation was found between miR-200c expression in tumors or plasma and clinical characteristics. Patients with higher miR-200c expression had better treatment outcomes with platinum chemotherapy and longer progression-free survival and overall survival than patients with lower miR-200c expression. Receiver-operating characteristic curve analysis showed that miR-200c expression in gastric cancer tissues and plasma distinguished patients’ treatment outcomes. Multivariate analyses confirmed that over expression of miR-200c both in gastric cancer tissue and plasma is associated with longer progression-free survival and overall survival. Taken together, our study indicated that miR-200c expression in gastric cancer tissues and plasma of patients with advanced gastric cancer is associated with better treatment efficacy and prognosis with platinum chemotherapy, suggesting that expression of miR-200c may be predictive for chemotherapy and prognosis in advanced gastric cancer patients.

## INTRODUCTION

Gastric cancer is the third leading cause of death in males and the fifth leading cause of death in females worldwide [1]. Although radical surgery is the most effective treatment,40–70% of patients are diagnosed with inoperable gastric cancer [2]. In addition, 40–60% of patients have recurrence after surgery [3, 4]. Five-year survival of advanced gastric cancer is only 5–20%, with the median survival time being less than one year [5, 6]. Platinum-containing chemotherapies are first-line treatment regimens for advanced gastric cancer but it is effective in only 29–48% of patients due to primary and secondary resistance [7–9]. Thus, there is an urgent need for better strategy for gastric cancer treatments.

Studies indicate that microRNAs (miRNAs) are involved in tumor formation, growth, and metastasis and can act as tumor suppressors or oncogenes. As biomarkers, they can be used for cancer diagnosis and predicting treatment outcomes and patient prognosis [10, 11]. MiRNAs are endogenous small non-coding RNA molecules of approximately 20–22 nucleotides in length. Through post-translational binding to complementary nucleotides in the 3’-non-coding region of target messenger RNA, miRNAs regulate target gene expression post-transcriptionally by inducing messenger RNA degradation or translation inhibition. MiRNAs can be released to plasma from normal or tumor tissues, and expression of miRNA in serum and plasma is relatively stable [12].

To minimize the invasiveness of biopsy collection and patient suffering, miRNA expression in tissue(s) can be predicted by measuring miRNA in plasma. Studies show that abnormal expression of miRNA is closely associated with the sensitivity of anti-cancer chemotherapy [13]. Therefore, miRNAs could be promising prognostic markers with predictive values for efficacy of chemotherapy [13]. Previous work indicated that miRNA-200c (miR-200c) expression in a cisplatin-resistant SGC-7901/DDP gastric cancer cell line was significantly lower than in the parental SGC-7901 cell line [14]. It was reported that the plasma levels of miR-200c emerged as an independent prognostic indicator for the survival of gastric cancer patients [15, 16]. To follow up these findings, we evaluated the association between miR-200c expression and treatment efficacy of first-line platinum-containing chemotherapies in patients with advanced gastric cancer. We also assessed the correlation of miR-200c expression in plasma and gastric tumor tissues.

## RESULTS

### miR-200c expression in advanced gastric cancer

The expression of miR-200c was evaluated in advanced gastric cancer and pericancerous tissues. As shown in Figure 1A, miR-200c expression in gastric cancer tissues was significantly lower than in pericancerous tissues (0.063 ± 0.021; 0.100 ± 0.019; *Z* = −5.755, *p<*0.05). Similarly, the miR-200c expression in plasma of patients with advanced gastric cancer (0.065 ± 0.034) was significantly lower than that in patients with chronic superficial gastritis (0.094 ± 0.020; *Z* = −4.155, *p<*0.05) as shown in Figure 1B.

**Figure 1:** Relative expression of miR-200c. (A) Relative expression of miR-200c in gastric cancer tissues and pericancerous tissue The expression of miR-200c is significantly lower in the gastric cancer tissues compared to tumor-adjacent tissues (*p<*0.05). **(B)** Relative expression of plasma miR-200c in patients with advanced gastric cancer and chronic superficial gastritis. The expression of miR-200c is significantly lower in patients with gastric cancer compared to those with chronic superficial gastritis (*p<*0.05) **(C)** miR-200c expression in tissue was positively correlated with that in plasma (Pearson's correlation coefficient *r*= 0.873, *p<*0.05; r^2^ = 0.762, Linear correlation analysis)

A linear correlation analysis of miR-200c expression in gastric cancer tissues and plasma was performed. As shown in Figure 1C, miR-200c expression in cancer tissues was positively correlated with that in plasma (Pearson's correlation coefficient *r*= 0.873, *p<*0.05; r^2^ = 0.762), suggesting that the expression of miR-200c in patients’ plasma could represent its expression in gastric cancer tissues. This result provided a rational for measuring miR-200c expression in plasma instead of cancer tissue, which is easier to perform in practice.

### miR-200c expression and treatment outcomes

Patients with efficacy assessments of CR+PR were categorized as having effective chemotherapy outcomes, and patients with results of PD were categorized as having ineffective treatment outcomes. Among those with advanced gastric cancer tissues and assessable chemotherapy efficacy, 11 had effective treatment outcomes and 17 patients had ineffective treatment outcomes and 23 patients were in stable condition. Relative miR-200c expression in advanced gastric cancer tissues of patients with effective chemotherapy(PR) outcomes (0.129 ± 0.026) was significantly higher than for patients with ineffective outcomes(PD) (0.060 ± 0.034) (*Z* = 5.749, *p<*0.05, Figure 2A). Plasma miR-200c expression is also related to treatment outcome. Relative plasma miR-200c expression for patients with effective chemotherapy outcomes(CR+PR) (0.112 ± 0.010) was significantly greater than for patients with ineffective outcomes (PD)(0.044 ± 0.026) (*Z* = 9.729, *p<*0.05, Figure 2B).

**Figure 2:** Expression of miR-200c and treatment efficacy in patients with advanced gastric cancer after platinum-containing chemotherapy Expression of miR-200c in gastric cancer tissue **(A)** and in plasma **(B)** of patients with treatment outcomes. There is a significant difference in patients with effective and ineffective treatment outcome (p<0.05, unpaired t-test).

### Association of miR-200c expression with patient clinical features and platinum-containing chemotherapeutic treatment efficacy

As shown in Table 1, miR-200c expression in advanced gastric cancer tissues and in plasma were not correlated with patients’ age, sex, ECOG score, tumor location, tumor tissue differentiation or liver metastasis (*P*> 0.05).

**Table 1:** Clinicopathological characteristics and miR-200c expression in gastric cancer tissues and plasma

Characteristics	Number	Percentage (%)	2^-ΔCt^ [X ± S](gastric cancer tissue)	P (gastric cancer tissue)	2^-ΔCt^ [X ± S] (plasma)	P (plasma)
**Gender**				0.714		0.951
**Male**	32	62.7	0.080 ± 0.040		0.064 ± 0.034	
**Female**	19	37.3	0.085 ± 0.040		0.065 ± 0.035	
**Age (years)**				0.145		0.229
**≧70**	16	31.4	0.070 ± 0.038		0.056 ± 0.033	
**<70**	35	68.6	0.087 ± 0.040		0.069 ± 0.034	
**ECOG (scores)**				0.402		0.934
**1**	40	78.4	0.084 ± 0.040		0.065 ± 0.034	
**2**	11	21.6	0.073 ± 0.040		0.064 ± 0.037	
**Differentiation**				0.362		0.309
**Poor**	32	62.7	0.078 ± 0.039		0.061 ± 0.032	
**Moderate and well**	19	37.3	0.088 ± 0.042		0.071 ± 0.037	
**Liver metastasis**				0.953		0.781
**Present**	21	41.2	0.082 ± 0.039		0.063 ± 0.036	
**Absent**	30	58.8	0.082 ± 0.041		0.066 ± 0.034	
**Tumor location**				0.801		0.406
**Proximal**	35	68.6	0.081 ± 0.043		0.062 ± 0.035	
**Distal**	16	31.4	0.084 ± 0.034		0.071 ± 0.031	

Platinum-containing chemotherapeutic treatment efficacy was evaluated in all 51 patients with advanced gastric cancer. There were 11 cases of PR, 23 cases of SD, and 17 cases of PD, with an objective response rate (ORR) of 21.6% and a disease control rate (DCR) of 66.7%. Relative miR-200c expression in cancer tissues was positively correlated with treatment efficacy (Spearmen's rank correlation coefficient *r_s_* = 0.581, *p<*0.05). ROC curve analysis was used to confirm the optimal threshold for prediction of disease control after chemotherapy, with an AUC of 0.751 and 95% confidence interval (CI): 0.605–0.897. When the maximum Youden index value was 0.382, relative miR-200c expression was 0.067, suggesting a sensitivity and specificity of platinum-containing chemotherapy for disease control of 0.676 and 0.706, respectively (Figure 3A).

**Figure 3:** ROC curve of miR-200c expression **(A)** The area under the ROC curve using miR-200c in gastric tumor tissues is shown [AUC 0.751 (95% confidence interval (CI): 0.605–0.897); cutoff value is 0.067; sensitivity, 67.6%; specificity, 70.6%]. **(B)** The area under the ROC curve using plasma miR-200c is shown [AUC 0.771 (95% confidence interval (CI): 0.640–0.902); cutoff value is 0.041; sensitivity, 76.5%; specificity, 64.7%].

Relative plasma miR-200c expression was also positively correlated with chemotherapeutic efficacy (Spearmen's rank correlation coefficient *r_s_* = 0.670, *p<*0.05). ROC curve analysis determined the best cutoff value for the prediction of disease control after chemotherapy, with the AUC of 0.771 and 95% CI: 0.640–0.902. When the maximum Youden index value was 0.412, relative plasma miR-200c expression was 0.041, suggesting a sensitivity and specificity of platinum-containing chemotherapy for disease control of 0.765 and 0.647, respectively (Figure 3B).

### Prognostic significance of miR-200c levels

After 13 months of follow-up, only 2 of 51 patients with advanced gastric cancer survived. All patients were divided into two groups based on median miR-200c expression in paraffin-embedded gastric cancer tissues. 26 cases had high expression of miR-200c and the median PFS was 5.9 months and 95% CI:5.0-6.8, median OS was 11.2 months and 95% CI:10.8-11.6). 25 cases had low miR-200c expression and the median PFS was 3.2 months and 95% CI: 0.8-5.6, median OS was 9.1 months and 95% CI:8.8-9.4. These results indicated that those with high miR-200c expression had longer PFS and OS (log-rank: *p<*0.05). Figure 4A and 4B depict survival curves of both groups.

**Figure 4:** Prognosis of miR-200c for gastric cancer patients treated with platinum-containing chemotherapies **(A** and **B)** patients with high level of miR-200c in gastric cancer tissue had longer PFS and OS than those with low miR-200c expression by Kaplan-Meier method (curves were separated by median value of miR-200c,both P<0.01) **(C** and **D)** patients with high plasma level of miR-200c had longer PFS and OS than those with low miR-200c expression by Kaplan-Meier method (curves were separated by median value of miR-200c,both P<0.01)

MiR-200c expression in plasma is associated with patients’ PFS and OS as well. The 51 advanced gastric cancer patients were divided into two groups based on median plasma miR-200c expression. Similarly, 26 patients had high plasma miR-200c expression and the median PFS of 5.9 months and 95% CI:4.9-6.9, median OS was 11.2 months and 95% CI:10.8-11.6. 25 patients had low plasma miR-200c expression and the median PFS was 3.2 months and 95% CI: 0.8-5.6, median OS was 9.2 months and 95% CI:8.6-9.8. Those with high plasma miR-200c expression had longer overall survival (log-rank: *p<*0.05). Figure 4C and 4D depict survival curves of the two groups.

Univariate Cox regression analyses revealed significant associations between expression of miR-200c both in tissue and in plasma as well as chemotherapeutic response and PFS (all p<0.001). The expression of miR-200c both in tissue and in plasma as well as chemotherapeutic response was also associated with OS (all p<0.001). Multivariate Cox model analysis demonstrated that expression of miR-200c both in tissue and in plasma and chemotherapeutic response are independent prognostic factors for PFS and OS (all p<0.05) (Table 2 and Table 3).

**Table 2:** Univariate Cox analysis of progression free survival and overall survival in gastric cancer patients

Parameters	Categories	HR(95%CI)	P value
PFS			
Age	≥70 VS <70	0.756(0.414-1.380)	0.362
Gender	Male VS Female	0.586(0.320-1.073)	0.083
Grade	G2 VS G3	0.796 (0.444-1.427)	0.443
ECOG	1 VS 2	1.370 (0.693-2.707)	0.365
Liver metastasis	Present VS Absent	1.103 (0.622-1.955)	0.737
Location	Proximal and body VS Distal	0.632 (0.338-1.184)	0.152
Chemotherapy regimens	Two drugs VS Three drugs	1.310 (0.708-2.422)	0.389
Chemotherapy response	CR+PR VS PD	0.007(0.001-0.066)	<0.001
	SD VS PD	0.015(0.002-0.132)	<0.001
miR-200c level(tissue)	High VS Low	0.217(0.105-0.449)	<0.001
miR-200c level(plasma)	High VS Low	0.244(0.120-0.496)	<0.001
OS			
Age	≥70 VS <70	0.812 (0.442-1.492)	0.503
Gender	Male VS Female	0.651 (0.362-1.170)	0.151
Grade	G2 VS G3	0.743 (0.414-1.332)	0.319
ECOG	1 VS 2	1.391 (0.703-2.752)	0.344
Liver metastasis	Present VS Absent	1.126 (0.632-2.006)	0.686
Location	Proximal and body VS Distal	0.504 (0.266-0.954)	0.035
Chemotherapy regimens	Two drugs VS Three drugs	1.582 (0.853-2.931)	0.145
Chemotherapy response	CR+PR VS PD	0.076 (0.029-0.196)	<0.001
	SD VS PD	0.152 (0.071-0.327)	<0.001
miR-200c level(tissue)	High VS Low	0.210 (0.105-0.420)	<0.001
miR-200c level(plasma)	High VS Low	0.292 (0.153-0.555)	<0.001

**Table 3:** Multivariate analysis of progression free survival and overall survival in gastric cancer patients

Parameters	Categories	HR(95%CI)	P value	HR(95%CI)	P value
PFS					
Chemotherapy response	CR+PR VS PD	0.012 (0.001-0.118)	<0.001	0.011 (0.001-0.113)	<0.001
	SD VS PD	0.020 (0.002-0.171)	<0.001	0.019 (0.002-0.166)	<0.001
miR-200c level(tissue)	High VS Low	0.350 (0.157-0.782)	0.01		
miR-200c level(plasma)	High VS Low			0.400 (0.182-0.877)	0.022
OS					
Chemotherapy response	CR+PR VS PD	0.105(0.036-0.305)	<0.001	0.102 (0.036-0.290)	<0.001
	SD VS PD	0.139(0.062-0.314)	<0.001	0.138(0.062-0.309)	<0.001
miR-200c level(tissue)	High VS Low	0.250(0.116-0.539)	<0.001		
miR-200c level(plasma)	High VS Low			0.356 (0.172-0.734)	0.005

## DISCUSSION

In this study, we demonstrated that miR-200c over-expression in advanced gastric cancer tissues and plasma was associated with better efficacy of platinum-containing chemotherapies and better clinical prognosis. Multivariate analyses confirmed that the level of miR-200c is independent prognostic factor. ROC curve analysis showed that miR-200c expression could be used to indicate chemotherapeutic efficacy. Importantly, miR-200c expression in gastric cancer tissue was positively correlated with that in plasma, suggesting that plasma miR-200c might be a potential molecular marker for predicting platinum-containing chemotherapeutic efficacy.

miR-200c is a member of miR-200 family, whose gene is localized on human chromosome 12 (12p13.31). Previously, high level of miR-200c expression was found in tumor tissue of some patients and associated with better prognosis [17]. It was suggested that miR-200c might inhibit epithelial-mesenchymal transition (EMT) to suppress the invasive and metastatic potential of tumors [18]. There were reports that miR-200c expression is related to tumor drug resistance. In some chemotherapy-resistant cancer cell lines (e.g., doxorubicin and cisplatin-resistant breast cancer cells and gemcitabine resistant pancreatic cancer cells), miRNA expression was significantly downregulated [19, 20]. Also, miR-200c directly regulates different targets to increase cancer cell sensitivity to microtubule-disrupted chemotherapeutic drugs and inhibitors of epidermal growth factor. Numerous solid tumor studies validated that tubulin-β3 (TUBB3) was involved in regulating the sensitivity of anti-microtubule chemotherapeutic agents (e.g., paclitaxel and vincristine) [21, 22]. miR-200c can directly target the 3’-UTR of TUBB3 mRNA, resulting in post-transcriptional suppression of TUBB3 expression [23], thereby improving sensitivity of paclitaxel, vincristine, and other drugs in tumor cells. Chen's group reported that miR-200c was associated with reversal of drug resistance, inhibition of SGC7901/DDP cell proliferation and induction of expression of E-cadherin, PTEN and BAX protein [14]. Finally, miR-200c was associated with activation of the Akt pathway and decreased expression of Bcl-2 protein [14]. Some published papers have claimed that gastric cancer patients have higher level of miR-200c expression than normal subjects and the miR-200c level was associated with certain clinicopathological characteristics including poor prognosis [15, 16]. This is different from our study and it may be due to different experimental design or sample size. Also, the above trials included patients with gastric cancer of all stages. Besides, not all patients received platinum-containing chemotherapies. Our study included only patients with gastric cancer at stages IV, and all the patients received platinum-containing chemotherapies. An article explains the discrepancies reported in the literature that analyzes the expression of miR-200c alone in ovarian cancer, claiming it as a marker of both poor and good outcomes [24]. HuR which is an RNA-binding protein, binds to multiple target mRNAs and regulates their stability and translation. It was reported that miR-200c exerted its influence to suppress TUBB3 gene/protein expression, when the HuR staining was found in nucleus, and as a consequence the tumor exhibited a good outcome. In contrast, the role of miR-200c appeared to be just the opposite when HuR localization was in cytoplasm. This phenomenon should be validated in gastric cancer.

To date, this study is the only clinical report suggesting an association between miR-200c over expression in tumor tissues and plasma are associated with better treatment outcomes with platinum-containing chemotherapy and better PFS and OS. miR-200c over expression was significant with respect in improving the prognosis of cancer patients. Due to short patient lifetime post-diagnosis, ineffective chemotherapy may increase suffering and diminish quality of life. Thus, miR-200c expression may be used to predict the efficacy of postoperative adjuvant chemotherapy to avoid ineffective chemotherapy and to prolong DFS. In addition, plasma expression of miR-200c was consistent with that in tumor tissues. Thus, plasma miR-200c expression could be used as a proxy of tumor tissue biopsy to predict efficacy of platinum-containing chemotherapy and to avoid tumor tissue collection in clinical practice. However, our study had some limitations such as a small sample size which may cause bias in the findings. Also, limited by gastroscopic tissue availability, we did not validate the molecular mechanism of miR-200c regulation.

In conclusion, we found that miR-200c over expression in gastric cancer tissues and plasma of patients with advanced gastric cancer is associated with better treatment efficacy with platinum chemotherapy and prognosis. MiR-200c could be a new biomarker for predicting treatment outcome and patient prognosis and guide the application of individualized medicine.

## MATERIALS AND METHODS

### Patients and specimens

Gastric cancer specimens were collected from 51 patients with advanced gastric cancer who received platinum treatment in the Department of Medical Oncology, the First Affiliated Hospital of Anhui Medical University, Anhui Province, China, from December 2014 to December 2015. Control patients were 51 subjects with chronic superficial gastritis diagnosed by gastroscopy. Patients with gastric cancer were confirmed by endoscopy or pathological examination after surgery and had to be at stage IV according to the AJCC/TNM staging system published in 2010. Patients should not receive chemotherapy or had the last chemotherapy >6 months prior to enrollment with measurable tumor lesion(s) by imaging. A lymph node must be more than 15mm in short axis and the longest diameter of the tumor lesions must be more than 10mm when assessed by CT or MRI scan. Patients also had to have a score ≤2 on the Eastern Cooperative Oncology Group (ECOG) scale of performance status; and had to have participated in at least two cycles of platinum-containing chemotherapy and had a follow-up with informed consent. MiR-200c expression in formalin-fixed paraffin-embedded gastric cancer tissue and tumor-adjacent tissues (gastric tissues ≥2 cm away from the tumor lesion) of all subjects was measured by qRT-PCR. In addition, plasma miR-200c expression was also measured by qRT-PCR before chemotherapy and compared to controls. Chemotherapy regimens included platinum (85 mg/m^2^ oxaliplatin d1 or 15 mg/m^2^ cisplatin d1–5) combined with fluoropyrimidine (2000 mg/m^2^capecitabine d1–14, 80 mg/m^2^tegafur/gimeracil/oteracil d1–14, or 400 mg/m^2^ 5-Fu iv d1 then 1200 mg/m^2^ lasting 24-h d1–2 combined with leucovorin d1, 400 mg/m^2^); taxane-platinum combination (135 mg/m^2^ paclitaxel d1 or 75 mg/m^2^ docetaxel d1); platinum plus fluorouracil-based chemotherapy with paclitaxel; platinum plus irinotecan (250 mg/m^2^ d1 irinotecan), repeated every three weeks (fluoropyrimidineand oxaliplatin regimen was repeated every two weeks). Chemotherapeutic efficacy was evaluated after two treatment cycles according to the standard of RESIST version 1.1, as four outcome measures, including complete response (CR), partial response (PR), stable disease (SD), and progressive disease (PD). Patients with efficacy assessments of CR+PR were categorized as having effective chemotherapy outcomes, and patients with results of PD were categorized as having ineffective treatment outcomes. CR+PR was used to calculate the objective response rate (ORR), and CR+PR+SD was used to calculate the disease control rate (DCR). Progression-free survival (PFS) was measured as the time between the baseline plasma sampling and the documentation of first tumor progression, based on clinical and radiological findings, or death (events). Overall survival (OS) was measured from the time at which the baseline plasma sample was obtained to the date of death from any cause or date of last follow-up. The patients who were alive and progression free at the time of analysis were censored by using the time between the plasma assessment and their most recent follow-up evaluations.

### RNA extraction from paraffin-embedded tissues

Two to three paraffin-embedded tissue sections (10-μm thickness) per sample were placed in a pre-labelled RNase-free Eppendorf (EP) tube, followed by the addition of 1 ml xylene solution. The mixture was vortexed for 10 s and centrifuged at 16,000g at room temperature for 2 min. The supernatant was discarded. Tissue pellets from each sample were washed with 1 ml of 100% ethanol, followed by centrifugation at 16,000 g, at room temperature, for 20 min and the supernatant was discarded again. After the pellet was air-dried at room temperature, 150 μl of proteinase K digestion buffer was added, followed by vortexing and mixing, and 10 μl proteinase K was added into the mixture and gently mixed. The mixture was incubated at 56°C for 15 min and subsequently at 80°C for 15 min. After incubation, the mixture was incubated on ice for 30 min, followed by centrifuging at 20,000 g for 15 min and the supernatant was transferred into a new EP tube. Sixteen microliters of DNase enhance solution and 10 μl of DNase I were gently mixed with the supernatant, followed by a brief centrifugation and incubation at room temperature for 15 min before mixing with 320 μl RBC lysis buffer and 1,120 μl 100% ethanol.

A 680 μl mixture was placed in a filter column, followed by centrifugation at 10,000 g for 20 s and the filtrate was discarded. This step was repeated until all sample mixtures passed through the filter column. Five microliters of RPE buffer was added to the filter column and centrifuged at 10,000 g for 20 s and the filtrate was discarded. A miRNeasy MinElute centrifugation tube was placed in a new collection tube and centrifuged at 14,000 g for 5 min. Filtrate was discarded and then the miRNeasy MinElute tube was placed in a new RNase-free tube, and 30 ul RNase-free water was added, followed by centrifugation at 14,000 g for 1 min. RNA purity was measured using aNanoDrop 1000 spectrophotometer. Those RNAs with the OD_260_/OD_280_ratio ranged from 1.8–2.1 were stored at a −80°C freezer and used for experiments.

### Plasma RNA extraction

Five milliliters of venous blood from each subject was collected in an EDTA anticoagulated tube and hemoglobin was measured to assure the quality of plasma sample for analysis of miRNA expression using a RNA extraction kit according to the manufacture's manual (Quiagen 74106). Spectrophotometry was used to assess the degree of hemolysis of plasma samples. If hemolysis occurred in the samples that were indicated by exceeding 0.2, then the plasma sample was excluded. Plasma samples with no hemolysis were centrifuged at 820 × *g*, 4°C for 10 min and the supernatant was carefully transferred into a new 1.5 ml RNase free EP tube and further centrifuged at 16,000 × *g* for 10 min. Collected supernatant was placed in a new 1.5 ml RNase free EP tube, which was stored at −80°C until used.

Four hundred fifty microliters plasma of each sample was placed in a new 2 ml RNase free EP tube after thawing, thoroughly mixed with same volume of 2× denaturing solution, and incubated on ice for 5 min before adding 900 μl phenol-chloroform solution. The mixture was vortexed for 20 s, and centrifuged at 12,000 g, room temperature for 5 min. Six hundred microliters supernatant were placed in a new 2 ml RNase free EP tube and added with 750 μl 100% ethanol and mixed thoroughly. Six hundred eighty microliters of the mixture were placed in a filter column, followed by centrifugation at 12,000 g for 30 s and the filtrate was discarded. This step was repeated until all mixture of the sample passed through the filter column. Seven microliters wash buffer 1 was added to the filter column and spun down at 12,000 g for 20s and the filtrate was discarded. Five hundred microliters wash buffer 2/3 was added to the filter column and spun down at 12,000 g for 20 s and the filtrate was discarded. The above step was repeated once. The filter column was centrifuged at 12,000 g for 1 min and added with 50 μl preheated elution solution (95°C water bath) before centrifugation at 12,000 g, room temperature for 1 min to obtain total RNA. A volume of 1.5 μl extracted RNA sample was used to measure the purity of RNA using a NanoDrop 1000 spectrophotometer. The ratio of OD260/OD280 should be ranged 1.8–2.1. Extracted total RNA was stored in a −80°C freezer for later experiments.

### Reverse transcription and qRT-PCR

Reverse transcription and qRT-PCR were performed according to the manufacture's manual (Biomics, Jiangsu Nantong). U6 siRNA was used as internal control in this experiment. The 25 μl qRT-PCR reaction system contained 3 μl total RNA extract, miR-200c- and U6-specific primers, forward and reverse primers, and 2× master mix. RNase-free DEPC water was used in the qRT-PCR reaction system. The prepared reaction system was placed in a PCR reaction strip, containing eight PCR tubes to start the qRT-PCR reaction in Mx300P qRT-PCR detection system. PCR conditions included reverse transcription at 42°C for 30 min; 95°C denaturation for 10 min; 40 cycles of 95°C denaturation for 20 s, 60°C annealing for 30 s, and 72°C elongation for 30 s. Fluorescent signals were collected at 72°C. The cycle threshold (Ct) value was defined as the number of cycles needed for the fluorescent signal intensity to cross the defaulted threshold in a quantitative PCR tube. Data were analyzed using ΔCt = Ct_miR-200c_− Ct_U6_ method. The 2^-ΔCt^ [13–14] represented the relative miR-200c expression in patients’ plasma and gastric cancer tissues. Each experimental sample was assessed in triplicate in three reaction tubes, and each experiment was repeated three times.

### Statistical analysis

SPSS17.0 software (SPSS Inc., Chicago, IL) was used for statistical analysis. Mann-Whitney U test was used for assessing miR-200c in gastric tissues and plasma. Prediction values of miR-200c expression in advanced gastric cancer for treatment efficacy of first-line platinum-containing chemotherapies were determined using receiver-operating characteristic (ROC) curve. The Kaplan-Meier method was used to prepare patients’ survival curves. Log-Rank test was used to compare the difference of survival curves of the two groups. The Cox proportional hazards model was applied to assess the correlations of the response predictor with PFS and OS.
